# Machine Vision-Based Ping Pong Ball Rotation Trajectory Tracking Algorithm

**DOI:** 10.1155/2022/3835649

**Published:** 2022-06-13

**Authors:** Yilei Wang, Ling Wang

**Affiliations:** ^1^Sports Department, Hangzhou Medical College, Hangzhou 310053, China; ^2^ZheJiang Gongshang University HangZhou College of Commerce, Hangzhou 311599, China

## Abstract

Because of the overwhelming characteristics of computer vision technology, the trend of intelligent upgrading in sports industry is obvious. Video technical and tactical data extraction, big data analysis, and match assistance systems have caused profound changes to all aspects of the sports industry. One of the important applications is the playback and analysis of sports videos. People can observe the videos and summarize the experience of sports matches, and in this process, people prefer the computers to also interpret and analyze sports matches, which can not only help coaches in postmatch analysis but also design robots to assist in teaching and training. In this paper, we have examined and designed an automatic detection system for ping pong balls, in which the motion trajectory and rotation information of ping pong balls are mainly detected. To achieve this goal, the detection and tracking algorithm of ping pong balls based on deep neural network is used, and better results are achieved on the data set established by ourselves and the actual system test. After obtaining the position of the ping pong ball in the image, the rotation direction and speed of the ping pong ball are calculated next, and the Fourier transform-based speed measurement method and the CNN-based rotation direction detection method are implemented, which achieve better results in the testing of lower speed datasets. Finally, this paper proposes an LSTM-based trajectory prediction algorithm to lay the foundation for the design of table tennis robot by predicting the trajectory of table tennis. Experimental tests show that the proposed system can better handle the ping pong ball tracking and rotation measurement problems.

## 1. Introduction

The objective of this work is to design a real-time accurate ping pong ball tracking system and to reconstruct the spatial coordinates of the ping pong ball using image information and camera position to calculate the ball velocity. In addition, the information and periodicity pattern of feature points on the table tennis ball in consecutive multiframe images are used to estimate the speed and rotation axis information of the table tennis ball and to extract the spatial position, speed, rotation axis, and other technical and tactical indicators of the table tennis ball. To test and perfect the whole system, it is necessary to measure and collect data in actual matches, measure the effect of the algorithm in actual table tennis match videos, and finally perfect the whole real-time table tennis analysis system. The research of this project includes the tracking system in table tennis matches, including target tracking and trajectory prediction for single-camera and two-camera systems, spin speed and rotation axis estimation of the ball, and visualization and analysis of the data. Combine traditional target tracking algorithms with the latest technologies to achieve a real-time table tennis match analysis system. The proposed model is developed based on these research objectives, i.e.,

- The design of a real-time accurate table tennis tracking system should be such that the reconstruction of the ball's spatial coordinates is carried out through image information and camera position. Similarly, these are used to calculate the velocity of the tennis ball as well.
- In consecutive multiframe images, the utilization of the information and periodicity pattern of feature points on the table tennis ball is for estimating its rotational speed and axis information.
- Collected data is visualized through the extracted spatial position, rotational speed, and rotation axis. Test and collect data in a real game, and improve the system.

In real-time accurate target tracking system, because of the small size, fast ball speed of table tennis balls, the presence of multiple interfering table tennis balls, and complex background effects in the actual game, it is common to lose the tracking target in the general tracking algorithm. By combining the background captured by the actual camera and the dynamic model of the ping pong ball movement, we build a new ping pong ball tracking system to achieve higher accuracy tracking while continuing to execute the target tracking algorithm once the tracking fails using the target recognition calculation to recalculate the position of the ping pong ball in the frame. For the other part, the algorithm that can estimate the rotation speed and rotation direction using the feature point information and period law of the ping pong ball on multiframe images requires estimating the three-dimensional spatial structure information on two-dimensional images using the spatial structure of the ping pong ball with the camera model. With the acquisition of sufficient amount of data, a visualization system for table tennis data analysis is built to facilitate players and coaches to get the needed information. The main contribution of this paper includes the following:

1. A migration learning-based target detection algorithm is proposed to detect ping pong balls, which combines coarse- and fine-grained features of the network to enhance its ability to match objects.
2. Additionally, we have proposed a deep neural network-enabled ping pong ball tracking algorithm to generate a probability map where the ping pong ball is located. Likewise, it generates the maximum connected component to output the final position and adds a wraparound box regression layer to refine the wraparound box coordinates to predict the correction value of the wraparound box. Finally, it outputs the wraparound box coordinates for each image frame, which is better in the tested.
3. To avoid the difficulty of reconstructing the spatial position of table tennis under dual viewpoints, this paper proposes an algorithm for recovering the spatial position of table tennis under single viewpoint, which uses the standard size of the table to calibrate the camera position. It also uses the size of the table tennis to calculate its spatial coordinates, which can be calibrated only once after assuming a good camera, and the algorithm dispenses with the problems of camera synchronization and high data transmission volume under multiple viewpoints. The algorithm eliminates the problems of camera synchronization and high data transfer under multiple viewpoints and is comparable in accuracy to that under dual viewpoints.
4. Two different types of ping pong balls are investigated for the measurement of rotational speed and spin direction. Firstly, an algorithm based on feature point matching and least square error estimation is proposed for logo balls to solve the optimal rotation matrix to obtain the rotation speed and direction of rotation. Then, to avoid the constraint of feature points, a Fourier transform-based rotation speed solution algorithm and a CNN-based rotation direction prediction model are proposed for logo balls and two-color balls.
5. An end-to-end LSTM-based trajectory prediction model is investigated and discussed. The model is designed with mixture density networks (MDN) to handle the ball bounce internally, which is integrated and tested with the whole system, and a large amount of video data is collected for experimental analysis and comparison.

The remaining portions or sections of the paper are arranged accordingly.

In Section 2, a brief but comprehensive study of the existing papers available in literature is presented, where it is particularly identified which issue is related with a particular scheme. In Section 3, we have discussed in detail our methodology, which has been presented in this paper to resolve the issue linked with the existing state-of-the-art approaches. As we have conducted experiments for the verification of the proposed methodology, its results along with detailed description are presented. Finally, concluding remarks are provided.

## 2. Related Work

With the improvement of computer processing performance and the development of computer technology, computer vision technology is playing an important role in more specific applications, one of which is in sports. For the general audience, the rich form of live streaming or broadcasting makes it is easier and higher quality for viewers to enjoy the game programs whether they are on or off the field. Secondly, for sports producers, computer technology can facilitate the organizers to monitor the games with commercialization prospects. In such a context, it is important to develop computer technology to support these application services. Technical and tactical analysis based on video understanding and motion tracking is an important research problem in the subject of sports video analysis. Sports video tactical analysis and motion analysis, on the other hand, are generally oriented to professional sports players and workers. Coaches and athletes can analyze sports videos to find their own athletes' shortcomings, learn other athletes' strengths, assist athletes' training, help teams specify tactics, etc. In addition, the tactical strategies behind the popular sports video games in recent years are also derived from the analysis of human game results, learning from the strategies of real games and applying them to the algorithms of virtual game characters. To achieve these goals, technical support is needed in many areas, such as computer vision, pattern recognition, and deep learning.

Existing sports video analysis systems include the Hawkeye system used in tennis [1] and the SportVU system equipped in professional basketball games in the United States. These systems are able to provide adequate data support to players and coaches using data analysis and visualization techniques while collecting large amounts of game data. In addition to recording statistics of lower-order data in sports, such as players' running distance and passing times in soccer games and assists and rebounds in basketball games, video data can be used to further analyze higher-order technical and tactical data, such as offensive plays [2] and blocking plays [3] in basketball games, etc. These systems and data analysis tools not only help coaches and players in their daily training but are also used in the broadcast of sports games, such as the technical and tactical review in live broadcast, all of which greatly enhance the viewing experience of the audience. This section will discuss the current state of research from different aspects.

### 2.1. Target Tracking

The target tracking problem is one of the most studied problems in the field of machine vision, and new techniques have been in development for decades. From traditional vision-based optical flow tracking, mean drift trackers [4], to later trackers integrating detection and machine learning, to today's deep learning-based tracking algorithms. Target tracking algorithms [5] are divided into two categories, namely (i) generative and (ii) discriminative, which depends on the modeling object. Generative methods model the current frame and determine those parts of distribution that are closest to the model prediction. The discriminative approach takes the parts containing the target as positive samples and other parts (e.g., background) as negative samples. It uses machine learning techniques to train classifier models by combining the local features of the image, such as the tracking learning detection (TLD) algorithm [6]. The discriminative approach considers background information, and therefore, it is more robust to background changes, whereas a majority of tracking algorithms are based on it.

Recently, correlation filter-based tracking algorithms have received more attention because of their speed, such as metaobject operating system environment (MOSSE) [7], CSK [8], KCF [9], and CN [10]. These algorithms learn a template to maximize the target's response to the template. This method changes the time domain correlation operation into a frequency domain dot product calculation by Fourier transform. Hence, it is fast, and then it outputs a response map by Fourier inversion back to the time domain, from which the coordinate information of the target is directly obtained. To increase the amount of data in the training template, the correlation filtering class method uses online learning to output a large amount of training data in a circular shift. The reason for it is that the samples obtained by densely sampling the vicinity of the target resemble the samples generated by circular shifting, and thus, they can be approximated by circular shifting. On the other hand, in terms of the angular aspect of the computation, convolution or correlation algorithms correspond to the dot product operations in the Fourier domain, and by converting the cyclic matrix to frequency domain diagonalization, combined with fast dot product operations can substantially reduce the computation time. Although the correlation filtering class of algorithms is fast, there are two problems that cannot deal well with the fast object deformation and fast motion situations. As filter correlation methods are generally based on template matching, once the object is deformed, then training template is invalid. Two types of deformation are used, i.e., if the shape changes rapidly, the gradient template based on the HOG feature is difficult to continue tracking. If the color changes rapidly, the color template based on the ColorName(CN) feature will fail. In addition, the parameters of the relevant filtering class methods are also difficult to determine. For example, assuming that the learning rate is updated by linear weighting, once the learning rate is too large, the model will learn the background information and will track the background area as time accumulates. Once the learning rate is too small, the template does not change in time after the target changes will also lead to tracking failure. Therefore, for the fast-flying ping pong balls in this paper, the correlation filtering class method has the advantage of speed, however, it is easy to follow the ping pong balls. TLD [6] (Tracking-Learning-Detection) is a representative of traditional tracking algorithms. It integrates the classical optical flow algorithm in computer vision, introduces ideas from target detection, and updates the tracker and detector with machine learning methods, and contains the basic modules of most modern tracking algorithms. The tracking module represents the object as a wraparound box and estimates the next frame of the wraparound box by estimating its displacement, deformation, and other parameters for the purpose of tracking. The detection module uses a sliding window to perform a full-image search and uses a classifier in machine learning to determine whether each window is a tracking target. The learning module is continuously updated using positive and negative examples for the tracking and detection modules, which also use P-N learning to ensure the effectiveness of learning. The quality of deep neural networks based on convolutional neural networks depends on the training of a large amount of data, and in the tracking problem, only the enclosing box of the target in the first frame is used as training data. DLT and others have adopted such an idea and used deep networks to directly replace the traditional manually selected features with good results, such as MDNet [11] and TCNN [12], in a real game of table tennis with fast ball speed and low camera. The low frame rate produces motion blur, resulting in unclear ping pong balls. Hence, higher frame rate cameras are often used in tournaments to achieve the condition of clear observation of ping pong balls. Hence, for using deep learning-based tracking algorithms, they need to be carefully designed to achieve the real-time requirements.

### 2.2. Rotation Measurement

Earlier, monocular vision systems were widely used [13, 14] as only one camera was used, and shadows were important for 3D ball localization. Therefore, such systems had restrictive requirements for lighting conditions and the speed and range of the ball flight. Recently, most table tennis robotic systems have used stereo vision systems and multivision systems [15, 16] to give more robust and accurate table tennis ball locations. Matsushima et al. [17] utilized a polynomial fit to estimate the ball state and two learned maps to forecast the ball's next trajectory. Zhang et al. [18] created a force analysis finding. According to Sun et al. [19], dynamic models can be described in both discrete and continuous versions, which share the same characteristics and are utilized for state estimation and trajectory prediction, respectively. They also presented a technique of learning and altering parameters to improve ball prediction at different flight speeds. This approach was successfully applied to humanoid robots, allowing them to play ping-pong continuously against each other or against human players. The algorithm mentioned above predicts the trajectory of a nonspinning ball very well but not for spinning balls.

Spin is a common occurrence while playing ping pong, and the trajectory prediction must consider the effects' information regarding the ball's spin. Based on the fast movement and high-speed rotation of the sphere in the flight of table tennis, a robotic vision system that can play table tennis against humans will be greatly beneficial to the development of high-speed visual perception, and the technologies involved for the recognition of the motion state of high-speed moving objects offer a wide range of industry application prospects, military, and other fields. The current algorithm for measuring table tennis rotation information is mainly obtained by the direct reduction of the feature point in the video in 3D coordinates and by tracking the trajectory of the point to calculate the coordinate changes in 3D. Russell Andersson's system is the first attempt to track the ball rotation. Since it only measured the rotation indirectly through the Magnus effect, the rotation was estimated with a lot of noise [20]. Fortunately, Andersson used only low-friction wooden paddles without a rubber surface, minimizing the effect of spin. Hence, the robot was able to play with moderate speed and spin against a crowd of people new to table tennis. Chen et al. [21], Huang et al. [22], and Su et al. [23] suggested that rotation could be estimated from trajectory deviations, and they used a motion pattern of the ball on the fly and a location vision system observed in flight trajectory. Calculate the force of deviation from the trajectory and then recover the rotation. Chen et al. [24] further demonstrated the bobbing system between the racket and the static ball, and by following the movement of the racket, they could ascertain how much revolution should be added to the static ball and use it to further develop the previous expected direction. Be that as it may, turn assessment dependent just upon position data includes a quadratic inference of position, which is exceptionally touchy to perception blunders, particularly assuming that the bearing of the pivot hub is like flight and heading and the rotational effect on the direction is tiny, then, at that point, a direction inclination-based approach would not be plausible. Their outcomes can give a reference to the heading of turn and the rough revolution speed. Yet, they are not sufficiently precise to empower the robot to hit a turning ball. Along these lines, a dream framework that can straightforwardly and precisely notice and gauge the revolution of a ping pong ball is required. Turn data improves the exactness of direction forecast, yet, in addition, it assists with better recreating the movement and skipping cycle of a turning ball. To get the twisted data straightforwardly, Boracchi et al. [25] gave a bunch of thoughts that can gauge the twist data of a ping pong ball from a solitary flight obscure picture. They re-enacted the camera imaging cycle to uncover the connection between the ball movement and the obscuring impact on the picture. This approach relies vigorously upon the picture nature of the ball and the markings ready surface, which restricts its application in table tennis games. Furuno et al. [26], Tamaki et al. [27], and Nakashima et al. [28] endeavored to quantify the ball turn utilizing UHF cameras (>600 outlines/sec). These cameras were mounted, keeping the optical line opposite to the heading of ball development. Hence, the picture size of the ball does not change a lot. To acquire a huge picture of the ball, the camera's field of view covers just a little piece of the flight way, which restricts its capacity to examine the whole direction. Theobalt et al. [29] utilized numerous openness pictures to recuperate the revolution of the ball. They directed tests in a dark indoor climate, where the screen and recurrence of the camera could be recreated by controlling the glimmer span and the recurrence of the light, and afterward, the 3D movement of the ball could be recuperated in the wake of getting numerous openness pictures of the whole flight. Watanabe et al. [30] used a multitarget tracking method to measure the rotation speed of the ball in real time using its unique features. The method first determines the 2D trajectories of multiple targets and then determines the 3D velocity vectors from the 2D trajectories. The velocity vector is used to obtain the rotation axis and rotation speed. However, this method requires a high frame rate vision system, and experimental results show that the measurable speed range is not adequate for table tennis matches. Liu et al. [31] pioneered a similar picture alignment-based speed estimation method by applying a ball rotation model to compare the picture data in a frame sequence. They used the least squares method to obtain the most reasonable rotational speed. Experimental results show that this method is accurate for a fast-flying ping-pong ball but has the same drawback as the previous method, i.e., a limited measurement range. Zhang et al. [32] attempted to construct the 3D coordinates of the ball directly and fit a plane with characteristic points to move the trajectory. They used the normal vector of the fitted plane to obtain information about the rotation axis and calculate the average rotation speed using the first and last positions of the feature points and the tracking duration. These vision systems mentioned above try to observe the spins directly, however, they all require specific lighting conditions and manually marked balls, which would change the physical properties of the balls and would not be allowed in a real game. In addition, their spin estimation methods depend heavily on the identification of the markers on the ball, and feature-based identification methods do not guarantee success rates. Therefore, human intervention is required. It limits the application of these methods in real-time broadcast tasks. Hence, this paper proposes a Fourier transform-based spin estimation method that avoids the drawback of requiring feature point matching.

## 3. Methodology

### 3.1. Deep Learning-Based Target Tracking Algorithm

#### 3.1.1. Background

Methods such as FCNT and CF2 have further explored the internal structure of CNNs and designed a more reasonable tracking framework. They found that the feature map of the convolutional layer in CNN can be used for tracking, and the feature maps of different layers have different roles in tracking. The feature map of the higher layer, which is closer to the classifier in the network structure, is good at distinguishing different classes of objects as well as robust in the deformation and occlusion of the target object, however, it is not able to distinguish different objects of the same class. The low-level feature map is more concerned with various local details of objects and can capture small differences between different objects of the same class. Moreover, since the pooling operation of CNN will downsample the upper layer, the closer the convolutional layer is to the input, the more position information can be retained, which is helpful for target localization during tracking. Specifically, FCNT extracts features from two convolutional layers with different depths for tracking to achieve a complementary effect. CF2 essentially adopts a correlation filtering approach. It trains three correlation filters from three convolutional layers. Each layer predicts a confidence map and improves the position prediction accuracy layer by layer. These methods combine the advantages of the layers within the CNN rather than just using the CNN as a black box, thus further enhancing the benefits of deep learning for target tracking problems. After this, more deep learning models think in terms of the nature of the tracking problem. Most of the above deep learning models are improved from image classification and detection tasks and are used as classifiers or detectors in tracking as well. Since only the first frame of the tracking task is an annotated sample, it is necessary to use the sample to retrain the above model and learn online in subsequent frames to make the tracking adapt to the current target. The literature [33] argues that the essence of target tracking is a verification problem, i.e., verifying whether the candidate region in the next frame is the same object as the currently tracked target. It is not classification or detection for a single frame. In [33], a special neural network structure is used to take two images as input and determine whether they are the same object. By giving the neural network this verification capability, the whole algorithm no longer relies on only labeled samples and online training. The literature [34] uses a similar network structure and completely discards the online learning part, enabling a deep learning-based tracking algorithm to reach 100 FPS for the first time.

#### 3.1.2. Algorithms

The target detection is intended to detect the desired object in a certain frame and mark it with a wraparound box. Hence, the detection technique often needs to detect the entire image range or use techniques, such as selective search, to detect the region proposal that may contain the target separately, which makes the whole process often time-consuming. Hence, directly apply the target to each frame of the video. The target detection algorithm is also often slow when applied directly to each frame of the video. This approach ignores the similarity and correlation between the front and back frames of the video, e.g., for a ping pong ball, there are shifts, size changes, texture changes, and light and dark changes in the front and back frames. However, the shape and color of the ping pong ball remain the same, and the texture changes periodically. We can assume that the rotation speed and direction of rotation of the ping pong ball remain the same during the flight. Hence, the changes of the logo pattern on the ping pong ball also show periodic changes. At the same time, the trajectory of the ping pong ball satisfies certain physical laws and is predictable before the ping pong ball hits the table. These factors are ignored in the target detection. Hence, it is necessary to process the target tracking module separately to efficiently track the trajectory of the ping pong ball.

Therefore, we want to implement a neural network for target tracking, in which the number of candidate images to be detected is as small as possible and the end-to-end output is achieved, i.e., the coordinates of the enclosing box containing the target are output directly instead of the feature vectors extracted by the convolutional neural network, thus simplifying the network structure and speeding up the computation.

The paper uses the tracking framework shown in Figure 1, where the input image is, firstly, deflated to the size of 100 × 100, and the final output is a 50 × 50 matrix, where each value in this matrix represents the probability that the pixels in the corresponding region of the grid belong to the tracking target. By setting a threshold, we make the probability map output a connected region, which completely represents the connected regions in the original input that belong to the target object and the probability values in the output connected. The probability value inside the connected region should be significantly larger than the part outside the connected region. The input image passes through a convolution layer and then a spatial pyramid pooling layer, so that the output layer contains more location information for each pixel with a larger perceptual field. In addition to the output target location, we have to do a binary classification to distinguish the target object from other background objects. Hence, our loss function is defined as follows:

(1) $$\begin{array}{c} L\left(p,s\right)=L_{\text{cls}}\left(s,s^{*}\right)+\lambda \sum_{i=1}^{50}\sum_{i=1}^{50}\sum_{j=1}^{50}-\left(1-t_{i,j}\text{log}\left(1-p_{i,j}\right)-t_{i,j}\text{log}\left(p_{i,j}\right)\right), \end{array}$$

where *p* and *s* are the output probability values and category scores, respectively, *s*^∗^ is the actual output category, *t*_*i*,*j*_ is the actual target probability map whether the target pixel is the target pixel, and *λ* is the regularization term to adjust the ratio of the two components.

The results obtained by this process are fast but not very accurate in the enclosing box for two reasons. Firstly, each pixel in the probability map corresponds to the size of the original 2 × 2 matrix. Hence, the judgment of the boundary part of the object is very rough. Secondly, the way to judge whether a pixel in the probability map belongs to the target object is by a simple threshold judgment, and the size of the ping pong ball will also change on the probability map with the change of distance from the camera. In the tracking process, if the bounding box is not accurate enough, the error will accumulate and the background pixels may occupy a large number of bounding boxes, leading to tracking failure until the target is lost. Here, we use a combination of coarse-grained features and fine-grained features similar to the target detection framework to perform wraparound box regression to correct the difference between the wraparound box and the actual target wraparound box. As shown in Figure 2, we add a region of interest pooling layer (ROI pooling layer), and we use the 23 × 23 × 96 low-level feature map obtained from the first convolutional layer as one of the inputs, which contains the low-level detail features as our coarse-grained feature input because it is closer to the input layer. The coarse-grained feature map is cropped and deflated to obtain a new 7 × 7 feature map, and then the coordinates of the enclosing box are regressed to output a final 4-dimensional vector, where the first two vectors represent the offset in the *x*, *y* direction and the last two represent the scale of *w*, *h*, which is in the range [0, 1]. The purpose of introducing the ROI pooling layer is to make the wraparound box coordinates closer to the target wraparound box position when regressing. Finally, we use the smooth L1 function as the loss function, which is defined as follows:

(2) $$\begin{array}{c} {\text{smooth}}_{L1}\left(x\right)=\left\{\begin{array}{cc} 0.5x^{2}, & \text{if}\left|x\right|<1,\\ \left|x\right|-0.5, & \text{otherwise}. \end{array}\right. \end{array}$$

By doing so, we use L2 loss near the origin and L1 loss in the rest to avoid the gradient explosion problem. We can get more accurate results by fine-tuning the probability map results using the enclosing box coordinates after the regression, and the specific experimental results and training steps are described later.

## 4. Experimental Results and Analysis

In this paper, we use Intel Core i7-4790K CPU, GeForce GTX1060 GPU, 6 GB video memory, 16 GB DDR3 memory, and Ubuntu 16.04 environment to implement and debug algorithms using the Pytorch framework and compare the differences of different algorithms. Pytorch is an open-source Python machine learning library that supports tensor computation on fast GPUs and makes it easy to write deep learning networks in the form of object-oriented programming, which supports automatic differentiation systems for backpropagation and updating network weights. In addition, with the visualization tools provided by tensorboard in tensorflow, it is easy to train, debug, and visualize deep neural networks.

### 4.1. Dataset

Whether it is a target detection or tracking algorithm, a large amount of labeled image or video data is required to train a deep neural network or to evaluate the performance of the algorithm, for which the preparation of data is the basis of the algorithm. “YouTube - 8M” [35] is a large labeled video dataset consisting of millions of YouTube videos, which contains thousands of videos ranging from 2 to 5 minutes in length from “Table tennis [2538],” as shown in Figure 3.

Although these videos are of high definition, the small size and fast motion of the table tennis balls make it difficult to apply these game videos directly to the detection and tracking of table tennis balls, as shown in Figure 4. It shows the blurred motion of the table tennis balls in the crawled video. The blurred request in the image leads to the tracking and detection algorithm to track incorrectly, and the detected enclosing box is difficult to determine the spatial location of the table tennis balls. The reasons are summarized as follows:

1. The motion blur caused by the low frame rate of the captured video leads to the inability to detect the specific location of the ball.
2. The clarity of the captured video is not high enough, and the noise is high enough to make it indistinguishable.
3. The camera is far away from the table, resulting in smaller and less detailed ping pong balls that cannot be tracked.
4. Even if the above conditions are satisfied, the lack of accurate labeling leads to errors in the model trained by the algorithm.

Therefore, we prepare the data by eliminating the images or video data that do not satisfy the above conditions. The process of preparing] the data is as follows: the video includes a constant speed serve with a tee machine and a multitap back and forth part of a two-person table tennis practice. The video with the tee machine is about 3s long, with a black cloth in the background to distinguish it from the white ping pong ball, which is less difficult. The video of two people practicing ping pong has no additional background treatment, however, there are no additional objects in the background, making it a little more difficult. Finally, we used a cell phone to shoot a video of a table tennis match, in which the background is complex and the most difficult. The different settings of the scene are shown in Figure 5. The data source for training the target detection algorithm is divided into two parts. There are unlabeled pictures of table tennis balls in ImageNet, which are downloaded and labeled using the auxiliary program written for the pictures. In addition, the ping pong ball position in each frame is, firstly, labeled from the directly captured video, and then, it is randomly cropped to generate images and add noise to generate more data, which partly includes ping pong balls and partly does not, for training the target detection algorithm, which eventually generates about 4000 positive sample images and 4000 negative sample images.

### 4.2. Experimental Results of Detection Module

Firstly, we discuss the selection of parameters for the training model, batch size = 128, momentum = 0.9, and decay = 0.0005, where the learning rate setting is special, as shown in Figure 6. Too high learning rate leads to large training error. Hence, we use 10-2 training 50 epochs at the beginning, then reduce the learning rate to 10-3 training 30 epochs, and finally train with 10-4. In this way, the convergence is guaranteed under the condition that the training speed is accelerated.

To avoid overfitting, the dataset is augmented using data augmentation, such as randomly scaling and panning the original image by no more than 20% of the original image size, adding random noise to the image, converting the image from RGB space to HSV space, and adjusting saturation and brightness. In addition, after we add a dropout layer to the first fully connected layer, we set dropout_rate = 0.5 to avoid coadaption between network layers, i.e., to avoid the phenomenon that the whole neural network depends on a few neurons.  Figure 7 show the variation of the training error with epochs and the model converges after 500 epochs.

To examine the role of migration learning, we compared the difference in precision (accuracy) and training time between Tiny Darknet as a pretrained network model and a randomly initialized model as a benchmark. As Figure 8 shows the variation of accuracy with training epochs, it can be seen that the accuracy of the pretrained network model is higher than that of the model without migration learning because the pretrained model is already better at extracting features.

Table 1 further describes the number of epochs that the model converges, the time required for each training epoch, and the total training time. The experimental results show that there is little difference in the average training time per epoch, as the pretrained model is used. Hence, the convergence is faster, and thus, the total training time is shorter.

### 4.3. Comparison of Target Tracking Experiments

#### 4.3.1. Performance Analysis

In this section, we analyze the performance of the proposed CNN model through experimental comparison, and we start from the following three aspects:

1. To judge the accuracy of the tracking module classification, we use the classification accuracy rate as the index.
2. To judge the accuracy of the output wraparound box, we compare the IoU to determine the degree of overlap between the wraparound box and the target.
3. To ensure real-time performance, the execution time of each part of the algorithm is measured.

To easily compare the advantages and disadvantages of this algorithm with other algorithms, a new model is trained based on the classical VGGNet-16. VGGNet has deeper layers than CaﬀeNet, and thus, it can learn higher-level semantic features. In general, the deeper the neural network, the better its ability to learn features and the better it is to classify them. VGGGNet-16 used in this paper consists of 13 convolutional layers divided into five groups. Each group of convolutional layers is followed by a 2 × 2 pooling layer, and the same ROI pooling layer is used as our network. The input feature map size is 50 × 50. Hence, the accuracy of the regression layer is higher compared with the algorithm in this paper. However, since the VGGNet network is deeper, the running time is significantly longer, and the training is more difficult.

Firstly, this section compares the accuracy of the tracking module, as shown in Table 2. Both models achieve high classification accuracy, with VGGNet being slightly more accurate because of its more powerful feature representation capability.

Secondly, Table 2 measures the difference in IoU scores before and after using wraparound box regression, and it can be seen from the table that the added wraparound box regression is more helpful in improving the location accuracy, while VGGNet scores higher than CaﬀeNet without or with regression layers. Next, we try to generalize the model used in this paper for tracking the ping pong balls to evaluate its ability as a general tracking framework.

Firstly, we compare the success plot and the accuracy plot, as shown in Figure 9. The success curve describes the relationship between the success rate and the set threshold during tracking, and it is defined as successful if the overlap between the predicted and actual wraparound boxes is greater than a given threshold. The success rate is, therefore, the percentage of the total number of frames tracked that are successful. The larger the threshold value set by the general tracker, the lower the tracking success rate. Ideally, we want the tracking success rate to be as high as possible with a high threshold value. Hence, we can calculate the AUC value (area under curve) of this curve to portray this property, AUC indicates the area wrapped by the curve, and a higher value indicates a better performance of the ping pong tracker. The accuracy curve describes the variation relationship between the accuracy rate and the set threshold value. If the distance between the predicted target position and the actual position at a certain moment is less than a certain threshold value, it is defined as tracking accuracy. Therefore, the accuracy rate can be defined as the percentage of the number of frames tracked accurately to the total number of video frames. The accuracy of the tracked target determines the accuracy of the subsequent spatial coordinate recovery, trajectory prediction, and other algorithms. Hence, it is the basis of the whole table tennis system and is a very important performance indicator. We choose the accuracy@20 with a threshold of 20 to measure the accuracy of the tracker and experimentally test the comparison using different CNN models. From the results in Figure 9 and Table 3, we can find that the VGG model outperforms the CaﬀeNet model. In the actual test, it can be found that the CaﬀeNet model is more likely to have a bounding box that does not fully include the target object, making the search box larger, and thus losing the target. Finally, we compare the differences between traditional target tracking algorithms, other deep convolutional network-based tracking algorithms, and our model. We implemented a color feature-based CamShift algorithm as the traditional tracking algorithm and used DLT and CF2 as the deep learning algorithms, and the experimental results are shown in Figure 10. The traditional method requires a high background, which can lead to tracking failure if there are background interferences, and the predicted bounding box is not accurate enough. Hence, we need to use methods, such as background rejection. Therefore, it is necessary to use methods, such as background rejection, to assist. The algorithm based on deep learning is more stable and less susceptible to background interference.

## 5. Conclusion

In this paper, we have tried to resolve various problems and difficulties, which are linked with existing methods, for estimating table tennis sports. For the existing target detection models, specifically those with background rejection techniques, we propose an end-to-end deep learning detection algorithm. The deep learning technique is incorporated into the ping-pong detection for each frame of the video image, and the corresponding optimal bracketing box output is obtained for the next step of processing. To address the slow rate problem of traditional methods for tracking fast moving objects, the proposed model achieves better real-time performance by simplifying the structure of neural networks for ping pong ball tracking and detection. After appropriate scaling of the image, each pixel point in the image is assigned a probability value belonging to the tracked object. The corresponding connected domains are judged and then input to the network for tracking judgment, and the tracking prediction results are quickly obtained. In response to the problems of the traditional multiviewpoint estimation of the spatial position of a ping pong ball, this paper proposes a single-viewpoint ping pong ball spatial position method. The final spatial position estimation of the ping pong ball is derived and optimized by presetting some a priori conditions, together with the motion of the ping pong ball in the actual problem, and verified by experiments. To address the problem that it is difficult to estimate the rotation of the ping pong ball itself in real situations, this paper proposes a classification analysis method based on feature color extraction and image superposition to estimate the rotational motion of the ping pong ball in combination with the corresponding CNN network. After extracting the ping pong ball, the image color is superimposed on the ping pong ball in consecutive frames, and the rotation frequency of the corresponding ping pong ball is obtained after fast Fourier transform.

## Figures and Tables

**Figure 1:** The architecture of tracking framework.

**Figure 2:** The architecture including ROI pooling layer.

**Figure 3:** You Tube-8M table tennis dataset.

**Figure 4:** Blurring in the video.

**Figure 5:** Video scenes.

**Figure 6:** The effect of various learning rates on training loss.

**Figure 7:** The training loss decreases as epochs.

**Figure 8:** The plot of precision vs epochs.

**Figure 9:** The left-accuracy plot. The right-precision plot.

**Figure 10:** Traditional tracking algorithm and deep learning-based tracking algorithm.

**Table 1:** Optimization of migration learning for training.

	Migration learning using Darknet-19	Without pretraining
Minimum epochs required for model convergence	510	960
Average training time per epoch (s)	36.52	38.52
Training time to converge (h)	5.17	10.24

**Table 2:** Comparison of classification accuracy and IoU scores.

	CaﬀeNet	VGGNet
Classification accuracy	0.985	0.997
Structured output CNN	0.512	0.618
Regression layer	0.713	0.611

**Table 3:** Target tracking metrics tested on the table tennis video dataset.

	CaﬀeNet	VGGNet
AUC	0.505	0.698
precision@20	0.877	0.971

## Data Availability

The data used to support the findings of this study are available from the corresponding author upon request.
